# Hand, Foot, and Mouth Disease in Thailand: A Comprehensive Modelling of Epidemic Dynamics

**DOI:** 10.1155/2021/6697522

**Published:** 2021-03-04

**Authors:** Suraj Verma, M. A. Razzaque, U. Sangtongdee, C. Arpnikanondt, B. Tassaneetrithep, D. Arthan, C. Paratthakonkun, N. Soonthornworasiri

**Affiliations:** ^1^School of Computing, Engineering & Digital Technologies, Teesside University, Southfield Rd, Middlesbrough, UK; ^2^King Mongkut's University of Technology Thonburi, Bangkok, Thailand; ^3^Center of Research Excellence in Immunoregulation, Research Department, Faculty of Medicine Siriraj Hospital, Bangkok, Thailand; ^4^Department of Tropical Nutrition and Food Science, Faculty of Tropical Medicine, Mahidol University, Bangkok, Thailand; ^5^College of Sports Science and Technology, Mahidol University, Nakhon Pathom, Thailand; ^6^Department of Tropical Hygiene, Faculty of Tropical Medicine, Mahidol University, Bangkok, Thailand

## Abstract

Hand, foot, and mouth disease (HFMD) is a highly contagious disease with several outbreaks in Asian-Pacific countries, including Thailand. With such epidemic characteristics and potential economic impact, HFMD is a significant public health issue in Thailand. Generally, contagious/infectious diseases' transmission dynamics vary across geolocations due to different socioeconomic situations, demography, and lifestyles. Hence, a nationwide comprehensive model of the disease's epidemic dynamics can provide information to understand better and predict a potential outbreak of this disease and efficiently and effectively manage its impact. However, there is no nationwide and comprehensive (i.e., the inclusion of reinfections in the model) model of HFDM dynamics for Thailand. This paper has endeavoured to promote nationwide comprehensive modelling of HFMD's epidemic dynamics and comprehend the reinfection cases. We have formulated the SEIRS epidemiological model with dynamic vitals, including reinfections, to explore this disease's prevalence. We also introduced periodic seasonality to reproduce the seasonal effect. The pattern of spread of this disease is uneven across the provinces in Thailand, so we used *K*-means clustering algorithm to cluster those provinces into three groups (i.e., highly, moderately, and least affected levels). We also analysed health records collected from district hospitals, which suggest significant reinfection cases. For example, we found that 11% (approximately) of infectious patients return for repeat treatment within the study period. We also performed sensitivity analysis which indicates that the basic reproduction number (*R*_0_) is sensitive to the rate of transmission (*β*) and the rate at which infected people recover (*γ*). By fitting the model with HFMD confirmed data for the provinces in each cluster, the basic reproduction number (*R*_0_) was estimated to be 2.643, 1.91, and 3.246 which are greater than 1. Based on this high *R*_0_, this study recommends that this disease will persist in the coming years under identical cultural and environmental conditions.

## 1. Introduction

HFMD is a paediatric disease that became an epidemic in the Asian-pacific region by the 1990s. This disease has spread in several Asian-Pacific countries, including Australia, Cambodia, China, Japan, Malaysia, Taiwan, Vietnam, and Thailand [1]. In Thailand, the first outbreak was recorded in 2012 with 45,464 infected people which was the largest in a decade. Thailand experienced the second outbreak of this disease in 2016 [2]. With such frequent outbreaks, HFMD has been a critical health issue in Thailand and has a tremendous socioeconomic impact. In addition to children's health, this disease affects their social life and education as they need to remain isolated from healthy children [3].

Though HFMD is a paediatric disease, even parents are affected as they have to take special care of their children during this period. HFMD outbreaks have caused a considerable economic strain in the affected nation's communities and healthcare systems.

Epidemic control agencies in Thailand have encountered many violent outbreaks that resulted in deaths. Despite being a common disease every year, it may not be diagnosed by a physician due to unclear appearances of rash [3, 4]. Many severe symptoms are misdiagnosed with a similar disease—encephalitis, pneumonitis, pulmonary oedema, or myocarditis. The outbreak of this virus in Thailand can be due to indirect transmission by environment infection, asymptomatic infected people, and patients who lack medical care [4]. Although serotyping is an immune response, a person can get HFMD more than once if they are infected with a different serotype [5].

Knowing a disease's (e.g., HFMD) current spread and forecasting the epidemic are significant for healthcare and financial planning. Mathematical models of epidemiology explaining the population dynamics of contagious diseases have played a significant role in the better understanding of epidemiological patterns and control of diseases [6]. The transmission patterns of infectious diseases vary through geolocations due to various socioeconomic conditions, demographics, and people's lifestyles [7]. Hence, a nationwide comprehensive model is required to understand the transmission of this disease.

There is no research that estimates the reinfection rate of HFMD in Thailand to the best of our knowledge. Also, no nationwide comprehensive epidemiological model has been developed to estimate the basic reproduction number (*R*_0_) for Thailand. In this context, this research is aimed at developing a nationwide comprehensive epidemiological model of HFMD in Thailand. The objectives of this research are (i) to estimate the reinfection rate of HFDM in Thailand, (ii) to identify and cluster the affected provinces of Thailand based on the severity of infection, and (iii) develop a nationwide comprehensive epidemiological model with dynamic vitals for those clustered provinces. We estimated the recurrence of HFMD from the data collected from three local hospitals in Thailand, and this estimated recurrence rate was considered in the epidemiological model. HFMD has an incubation period in the host before they become infected. The incubation period is when an individual is exposed to the virus but not yet infected. Therefore, we considered the SEIRS (susceptible-exposed-infectious-recovered-susceptible) model in this paper, which addresses both the reinfection cases and the incubation period of the disease. This model describes the spread of HFMD and estimates the infection rate, recovery rate, and the basic reproduction number. Also, periodic seasonality was introduced in the model to address the seasonal outbreaks, which occur every rainy season. The data of hospitalised patients collected from BoE National Disease Surveillance (report 506) [2] was used to fit the proposed model and estimate the basic reproduction number (*R*_0_). This paper describes the simulation of the proposed model and performs sensitivity analysis to analyse input parameters' impact in estimating *R*_0_.

Section 2 provides a brief literature review of related works conducted to estimate the basic reproduction number (*R*_0_) to understand HFMD disease transmission.  Section 3 presents the materials and methods, including data collection and preprocessing, construction of the theoretical SEIRS model, and sensitivity analysis. The results from the study of the collected data are summarised in Section 4. This section also discussed the results obtained from clustering and fitting the clusters in the model using *R*^2^ to check the goodness of fit. In Section 5, we discussed the findings from the analysis and case study performed and the impact of COVID-19 in the spread of HFDM. Finally, we conclude the work with potential future research direction.

## 2. Related Works

In epidemiology, there is a long history of mathematical models. Many epidemiological models like SIR, SEIR, SEIQR, SEIRS, and many other models have been introduced to estimate infection rate of contagious diseases. The majority of these models are compartmental models, where the population is divided into compartments/groups with an assumption that the population transfers from one compartment to another [8]. Several mathematicians and researchers have proposed various epidemiological models to understand the transmission of HFMD better. Chuo et al. [9] used a SIR model to predict the number of infected people during the outbreak of HFMD in Sarawak of Malaysia. However, this model did not consider any seasonality effect and reinfection cases to spread this disease. Later on, a periodic model considered with quarantine effect was proposed by Liu [10]. Du et al. [7] adopted another approach to model this disease using time-series susceptible-infected-recovered model. In this model, a time scale for this disease was considered two weeks based on the characteristics of HFMD where the duration of the transition from infection to recovered and temporary immunity is about 7 to 10 days.

Very few studies have been conducted for modelling the outbreak of this disease in Thailand. Chadsuthi and Wichapeng [4] researched the outbreak of HFMD in Bangkok in 2016 and proposed a customised SEIR model. The customised model considered susceptible (*S*), exposed but not yet infectious (*E*), infectious but with no symptoms (*I*_*e*_), infectious with symptoms (*I*), hospitalised (*H*), and recovered (*R*). The basic reproduction number (*R*_0_) was predicted to be 1.441. However, the study conducted was during the outbreak of 2016 for Bangkok only, and no seasonal effect was considered in this model.

Furthermore, in a study conducted by Huang et al. [11], it is found that multiple viruses, Enterovirus-71 (EV-71) and Coxsackievirus A16 (CA 16), are the causative agents of HFMD. Children infected with one virus are likely to be infected with other viruses that cause the same disease. As per their study conducted in China, 1.9% were reinfected at 12 months, 3.3% at 36 months, and 4.0% at 38.8 months. However, no study is taking care of the cases of reinfection in Thailand. Significantly, to date, no nationwide and comprehensive model has been developed for modelling the transmission of HFDM that considers seasonal effect and reinfection cases. CV-A16 and EV-A71 related to HFMD were analysed with an epidemic model in 2016 in China by [12]. Analysing time series then SIR modelling made this work having a model fit. Seasonality and heterogeneity were key features extracting from the province-level transmission. EV-A71 had a reproduction rate less than CV-A16, which was 26.63 and 27.13, respectively. Although their prediction was concentrated in sensitivity analysis, the primary purpose was to distribute vaccination effectively for herd immunity in a province, not to calculate the reinfection rate as we are proposing.

## 3. Materials and Methods

### 3.1. Data Exploration

For this study, we collected province-wise monthly reported data (from January 2011 to July 2020) of HFMD cases from BoE National Disease Surveillance (report 506) [2]. We also gathered data for HFMD cases for the different age groups of people in Thailand for 2019 from BoE. The population of children under 14 years for years 2019 was collected from the World Bank Group [13]. Moreover, to understand the reinfection cases, patients' records were collected from three local hospitals: Samut Sakhon, Suan Pueng, and Ranong. These are district hospitals that offer standard medical services for Thai and non-Thai residents. The local datasets were derived from a retrospective study associated with hospital patients' situation and trend in western borders between 2012 and 2016 [14]. All the personal identifiers were removed from the dataset to maintain the patients' privacy. The Faculty of Tropical Medicine at Mahidol University gave ethical approval for the retrospective analysis that obtained local datasets.

Data collection began with a selection of public-access health facilities. The sample involved the three public hospitals mentioned earlier. Service capabilities are similar to those of medical centres located in urban areas. For the study, we collected the patients' records admitted to each hospital between 2012 and 2016. As HFMD is a paediatric disease, we separated the under fifteen age patients' records for the study. The diagnostic statistics data was collected from the outpatient and inpatient medical record database. We used Equation (1) to identify the minimum sample size of the medical record required for our estimation [15].

(1) $$\begin{array}{c} n=Z^{2}pq/d^{2} \end{array}$$

where

- *n* is the minimum sample size needed for the study
- *Z* is the level of confidence according to the standard normal distribution. For example, for a level of confidence of 95% or 5% level of significance (*α* = 0.05), *z* = 1.96
- *p* is the prevalence of the disease in children
- *q* is a subcalculation with 1 − *p*, or percentage of failure
- *d* stands for precision limit or proportion of sampling error which is usually 5% confidence limit

From the experiment, it was found that the minimum number sample required for the estimation is 384. Patient data were collected from the Medical Record Program for Enterovirus Infectious Disease. The disease codes B08.4, B08.5, and K12.0 were randomly sampled to obtain at least 384 records.

### 3.2. Data Preprocessing

The first step was preprocessing and cleaning the raw data to fit into the model. We performed this operation in two steps. First, we preprocessed the data to get HFMD cases across the provinces in Thailand, as shown in Figure 1. For this purpose, we built a data model from raw data of Thailand population, HFMD cases, and Thailand's provinces geocoordinates. The data was then cleaned by removing irrelevant, null, and empty data, and the cleaned data was transformed into the expected format. Finally, we extracted province-wise infected data and infection-wise health district zones. After getting the data for HFMD cases across different provinces in Thailand, the second step was to get the disease's reinfection rate in Thailand. For this purpose, we processed the raw data collected from three local hospitals:; Ranong Hospital at the southern border, Samut Sakhon Hospital at the central area, and Rachaburi at the western border in Thailand Figure 2. We compiled all the data and filtered the HFMD cases' data (ICD-10 code: B084). Then, patients' details were deidentified to maintain their privacy. To extract the patients who revisited the hospital with HFMD complaint, patients with a record count ≥ 2 were identified. Follow-up records were removed to get the revisit of HFMD cases but not a follow-up treatment.

### 3.3. Model

We modelled the trajectory of the infection of HFMD disease in Thailand for years 2011 to 2019 using the SEIRS model with vital dynamics, a compartmental model. The incubation period of the disease is considered in this model [16]. This model also addresses the reinfection cases where a fraction of the recovered patients get reinfected with the same disease. The population is divided into four compartments, as shown in Figure 3. The compartments are represented by *S*, *E*, *I*, and *R* where

- Susceptible (*S*) denotes people who are not infected but can get infected
- Exposed (*E*) denotes people who are exposed but not yet infected
- Infected (*I*) denotes people who are infected and can pass it on
- Removed (*R*) denotes people who have recovered from this disease or died

Let us assume the total population of children who can be infected with HFMD by *N*. Then, the total population can be represented as, *N* = *S* + *E* + *I* + *R*. The equations for the SEIRS model are as follows:

(2) $$\begin{array}{c} \frac{dS}{dt}=\mu \left(N-S\right)-\beta \frac{I}{N}S+\omega R,\\ \frac{dE}{dt}=\beta \frac{I}{N}S-\left(\sigma +\mu \right)E,\\ \frac{dI}{dt}=\sigma E-\left(\gamma +\mu \right)I,\\ \frac{dR}{dt}=\gamma I-\left(\mu +\omega \right)R. \end{array}$$

Here, *μ* represents the birth and mortality rates per capita. Let us assume that the birth rate and the death rate are the same, giving the constant population throughout the year. *β* represents the contact/transmission rate at which infected individuals contact susceptible people to spread the disease. If*I*is infected people, contact*S*is susceptible people, and the rate at which disease can spread is*β*, then *β*(*I*/*N*) S represents the average number of infections. 1/*σ* and 1/*γ* represent the mean latent period and infectious period, respectively. The rate at which recovered patients become susceptible is represented by *ω*. The basic reproduction number (*R*_0_) used to measure the transmission potential of this disease using this model is calculated by Equation (3). At the same time, 1/(*β* + *μ* + *α*) gives the infectious period and the probability index of becoming infectious rather than dying. *σ*/(*σ* + *μ*) gives the probability index of becoming infectious while exposed (*E*).

(3) $$\begin{array}{c} R_{0}=\frac{\beta }{\left(\sigma +\mu \right)}\frac{\sigma }{\left(\gamma +\mu \right)}. \end{array}$$

### 3.4. Seasonality of Transmission

HFMD in Thailand is a recurring epidemic disease. Historical data demonstrates that the disease outbreaks happen seasonally during the rainy season each year. The transmission rate varies seasonally giving a spike during the rainy season. The seasonal transmission was considered in our model, focusing on the transmission rate *β* as *β* = *β*(*t*). A sinusoidal trigonometric function was introduced to estimate *β* as follows:

(4) $$\begin{array}{c} \beta =\beta_{0}\left[1+\sin\left(\frac{2\pi \left(t+\alpha \right)}{T}\right)\right], \end{array}$$

where *β*_0_, *α*, *t*, and *T* represent the baseline of transmission rate, a time constant, time, and period of seasonal cycle, respectively [17]. The main advantage of introducing this trigonometric function is to explore the qualitative characteristics of seasonally varying disease transmission and variable transmission rate.

### 3.5. Sensitivity Analysis

To identify the parameters that influence the basic reproduction number (*R*_0_), we performed a sensitivity analysis of the model. We used python's SALib library to perform Sobol sensitivity analysis, a global sensitivity analysis [18]. First, the input parameters (beta, sigma, gamma, and mu) required to estimate the basic reproduction number to calculate the sensitivity were determined. Then, 1000 parameter samples were generated using the satellite library. Finally, the sensitivity index was calculated using the library's analysis function on the output function using samples. Three different types of sensitivity indices, first-order, second-order, and total-order index, were calculated. The first-order index (S1) measures the contribution of the individual input parameters to *R*_0_. The second-order index (S2) measures a contribution of the combination of two parameters to *R*_0_. Similarly, the total-order index (ST) measures the contribution of both first- and higher-order indices on *R*_0_.  Table 1 provides the details of the first-order and total-order sensitivity index of parameters on *R*_0_. It is seen that the first-order and total-order indices for beta and gamma are much higher compared to those for sigma and mu, indicating that these parameters are highly influencing parameters for the estimation of *R*_0_.  Table 2 provides the details of the second-order sensitivity index for the combination of parameters. Here, a combination of beta and gamma has a higher value for the second-order index, indicating that these two parameters are crucial for calculating *R*_0_.  Figure 4 illustrates the influence of each parameter on the basic reproduction number (*R*) for 1000 samples. As seen in the figure, we can determine that beta and gamma directly relate to the estimation of *R*_0_. For a grouped bar graph, Figure 5 was plotted to analyse the sensitivity of parameters. From this graph, it is seen that beta and gamma are critical parameters for *R*_0_. Although there is no cut-off value of sensitivity index, we considered the sensitivity index value > 0.05 as an important parameter for estimating *R*_0_. In the figure, the total-order index (ST) value greater than the first-order index (S1) value indicates that there are higher-order interactions.

### 3.6. Data Fitting and Mathematical Simulation

This study applies *K*-means, a self-adaptive weight clustering algorithm, to identify or cluster the provinces that are highly, moderately, and least affected with this disease to better estimate the basic reproduction number for those clustered provinces. The data collected from the BoE for the provinces in each cluster was fitted to simulate the SEIRS model. The initial values for *S*_0_ were taken as 3604225, 6563387, and 779287 for provinces in clusters 1, 2, and 3, respectively. Similarly, initial values for *E*_0_ and *R*_0_ were considered 0. The time of each cycle (*T*) was considered 12 months. The reinfection rate (*ω* = 0.119) estimated from the three local hospitals' dataset was also considered in our model. We used SciPy optimiser's curve fitting tool to fit the model with the data and estimate the parameters. The curve fitting tool uses the least-squares minimisation technique to fit the data in the model. The goodness of fit of the simulated model was estimated using the determination coefficient (*R*^2^).

## 4. Results

We analysed the collected data to understand the spread of HFMD in different provinces throughout the year. We found that the disease outbreak generally occurs in June, July, and August of each year throughout Thailand. Two outbreaks were seen in 2012 and 2016, where the number of infected cases during the rainy season was very high compared to other seasons (Figure 6). We plotted a heat map for HFMD cases to visualise the spread of this disease across provinces during the years 2011 to 2019. From the heat map, we found that, according to the severity of infections, the provinces could be grouped into three clusters (Figure 7). Thus, the *K*-means algorithm was applied to cluster the provinces based on the number of infection cases from 2011 to 2019. Based on the severity of infection of the disease as observed in the heat map and *K*-means clustering result, we identified three different clusters of provinces in Thailand. The provinces are clustered into highly, moderately, and least affected provinces, as shown in Figure 8 and Table 3.

To analyse the age group of infected people in Thailand, we plotted a bar graph for 2019. As expected, we observed that children under 14 years are more infected than older people (Figure 9).

The severity of infection of this disease across the provinces in Thailand was visualized by plotting a heat map over the provincial map of Thailand (Figure 10). We used “Paintmaps” online tool to plot the heat map over Thailand's provincial map and visualise the geographical spread of this disease for the year 2019. This geographical map illustrates that HFMD has spread in most of the provinces, and Bangkok is the most affected province. From the case study performed at three different local hospitals in Thailand, we found that a significant number of patients who visited the hospital were reinfected with HFMD. For the selected three hospitals (2012-2016), we found different cumulative reinfection cases or rates which are not insignificant, and it is increasing with the inclusion of an additional year (Table 4). For example, the reinfection rate or percentage for the year 2012-2015 is 9.39%, which has changed to 11.92%, adding the year 2016.

### 4.1. Fitting the Model

SEIRS model was fitted using curve fitting, and the goodness of fit of the model to the recorded data for each cluster is illustrated in Figures 11–13 for provinces in clusters 1, 2, and 3, respectively. The model fitted the HFMD models for the years 2011 to 2019. For better fitting, the model was fitted for each year, and values for the parameters *α*, *β*_0_, *σ*, *μ*, *γ* were estimated.

### 4.2. Estimation of Parameters

For the model simulation, the value of *N* was considered the population of children under 14 years. The initial infected population, *I*_0_, was taken from the BoE. The parameters *α*, *β*_0_, *σ*, *μ*, and *γ* were estimated by fitting the recorded data in the model using curve fit. Tables 5–7 illustrate the estimated parameters for the provinces in clusters 1, 2, and 3, respectively. The tables also show the calculated basic reproduction number *R*_0_.

### 4.3. Validity of Model

The goodness of fitting of the model was tested by regression analysis. The determination coefficient (*R*^2^) was calculated using the following formulae (5), (6), and (7):

(5) $$\begin{array}{c} \text{S}{\text{S}}_{\text{tot}}=\underset{i}{\sum }{\left(y_{1}-\overset{\wedge }{y}\right)}^{2}, \end{array}$$

(6) $$\begin{array}{c} \text{S}{\text{S}}_{\text{res}}=\underset{i}{\sum }{\left(y_{1}-f_{1}\right)}^{2}, \end{array}$$

(7) $$\begin{array}{c} R^{2}=1-\frac{\text{S}{\text{S}}_{\text{res}}}{\text{S}{\text{S}}_{\text{tot}}} \end{array}$$

The standard of model fitting has been evaluated for each cluster independently by calculating *R*^2^ using Equation (7). The result for *R*^2^ obtained for each cluster model is illustrated in Table 8. The values are greater than 0.6 which illustrates that at least 60% of the recorded data fitted well in the model. Out of three clusters, for cluster 2, the model fitted the recorded data very well with *R*^2^ 77.7%.

## 5. Discussion

The major finding of this study is the reinfection rate of HFMD in Thailand. HFMD-recovered patients become immune to the virus, and the chances of getting reinfected with the same virus is scarce. However, as the disease is caused by multiple viruses (Enterovirus-71 (EV-71) and Coxsackievirus A16 (CA 16)) [19], there is a chance of getting infected with other virus causing the same disease. From the result of the case study performed at three local hospitals in Thailand, it is found that 11.92% (approximately) of the recorded cases are reinfection cases. The case of reinfection is significantly high, especially during the rainy seasons.

HFMD is most prevalent spreading in younger ages compared to the older groups of patients across the country. During the mid of each year, the total number of patients increases consistently in a similar previous pattern. One of the reasons is that the rainy season in Thailand starts from early May to late July and this disease transmits quite rapidly during the rainy season. Moreover, primary and secondary schools begin the first semester in the middle of May [20], which leads to an increase in physical contact between infected and susceptible children. At the beginning of the school term, children are not provided with full support, especially wellness and health checks and physical education. These may cause the infection to reach a peak during the mid of each year. The reinfection is also the supporting cause of outbreak during rainy seasons each year.

Figure 6 illustrates that the number of infected cases is very high during rainy seasons and the outbreak of this disease occurred in 2012 and 2016. The heat map (Figure 7) and geographical map (Figure 10) help us to visualise the spread of this disease across all the provinces. We found that all provinces are not equally affected. Bangkok is observed to be the most affected province. Since this disease's transmission is uneven across the provinces, it is essential to identify the provinces with similar disease severity. Hence, we utilised the *K*-means algorithm to cluster the provinces based on the severity of the infection cases. The resulting cluster grouped the provinces into three categories, highly, moderately, and least affected provinces. The main advantage of clustering the provinces based on the number of infections is that positively affected provinces can get more attention and the healthcare facilities and human resources can take appropriate actions to control the disease.

Mathematical models have always been an essential tool for understanding the spread of epidemiological diseases. No comprehensive model has been developed to address this disease's nationwide transmission with reinfection cases in Thailand. To understand and predict the spread of this disease, we have built a comprehensive compartmental SEIRS model with vital dynamics by incorporating the BoE surveillance data and reinfection rate estimated from the three hospitals to estimate the *R*_0_ of HFMD. We have also introduced periodic seasonality to address the seasonal effect in preventing this disease. Generally, the time from initial infection to the occurrence of signs and symptoms (incubation period) of HFDM is 3 to 7 days [19]. During this period, infected people are not yet infectious.

According to the proposed model, *E* (exposed) addresses the incubation (latent) period. This model also addresses the rate of reinfection where a fraction of the recovered patients become susceptible because of different virus type. *ω* is the rate at which recovered patients become susceptible. The proposed SEIRS model was fitted with recorded HFMD cases based upon each cluster's provinces to better estimate the parameters. Figures 11–13 illustrate the goodness of fit of recorded data for HFMD cases in provinces in clusters 1, 2, and 3, respectively. The model fitted well the outbreaks of this disease seen in the rainy season of each year. While fitting the model, *α*, *β*_0_, *σ*, *μ*, and *γ* parameters were estimated which are illustrated in Tables 5–7 for provinces in three clusters. The basic reproduction number (*R*_0_) obtained from the simulation of three clustered provinces is greater than 1, indicating that this disease will persist in the coming years under the same social and environmental condition.

HFMD is transmitted primarily through direct contact with contaminated discharge, saliva, or stool from infected patients or contaminated objects. Moreover, attending kindergarten or child-care centres or schools increases the risk factor for the transmission of this disease [21]. Avoiding physical interaction with infected people, such as kissing, embracing, and sharing cups and eating utensils, plays a significant role in minimising the spread of this disease. Because of the COVID-19 pandemic, a nationwide lockdown and quarantine of infected patients were imposed. The schools were closed, and no physical contact was made with infected patients which played significant role in reducing HFMD cases in 2020. For each month of this year, the number of infected cases was decreasing. The predicted number of HFMD-infected patients and the recorded number of cases for the year 2020 for each cluster are illustrated in Figures 14(a)–14(c). These figures illustrate a significant decrease in the number of infected cases. Even during the rainy season, the cases were decreasing because of the impact of COVID-19 lockdown imposed in the year 2020.

This study estimated the HFMD reinfection rate from limited data collected from three local hospitals in Thailand. This estimate could have been improved by collecting more and random samples from hospitals from different regions of the country or the Bureau of Epidemiology (BoE). However, due to the COVID pandemic, we could not collect sufficient data. Our model considers the reinfection rate for the estimation of the transmission rate (*β*), the recovery rate (*γ*), and the basic reproduction number (*R*_0_), so an improved reinfection rate estimate can improve the estimation of *β*, *γ*, and *R*_0_. Also, HFMD-infected patients may not show any symptoms but can still spread the disease. Such infections are asymptomatic infections. Many HFMD-infected patients are hospitalised, which reduces the physical contact between infected and susceptible patients. Thus, asymptomatic infections and hospitalisation cases are essential factors for estimating the basic reproduction number. However, due to the limited available data, these factors have not been considered in our model.

## 6. Conclusions

This paper has estimated the recurrence rate of HFMD disease in Thailand. We have applied the estimation to develop a nationwide and comprehensive model of epidemic dynamics using the SEIRS model. With dynamic vitals, including reinfections, our results indicate that this disease's transmission is most prevalent in midyear. From the experiment performed using the model and study conducted at three provincial-level hospitals, we can conclude that this seasonal disease is a critical health issue.

The spread of this disease is uneven throughout the provinces across the country. Hence, we clustered the provinces into three clusters based on the number of infections from the years 2011 to 2019 and the basic reproduction number (*R*_0_) obtained from the SEIRS model for all these clusters is greater than 1, which indicates that under the same social and environmental condition, this disease will persist in the coming years.

Moreover, we learned that the reinfection rate, especially during the rainy season, is remarkably high in Thailand. Such circumstance is one of the main reasons for higher infection rates or cases during the rainy season. However, the number of infected patients is significantly low for 2020 due to the COVID-19 pandemic. The lockdown imposed on account of the pandemic minimises direct or indirect physical contact with infected people and spread of COVID-19. This measure also helped to minimise the spread of HFMD. So, taking proper and informed actions could improve the management of HFMD-like diseases in Thailand and globally. Informed actions need real-time or quasi-real-time data about infected people. Hence, our future endeavours will focus on smartphone-based digital diagnosis and reporting of HFMD.

## Figures and Tables

**Figure 1:** Data collection and preprocessing steps for extracting data to fit into the model.

**Figure 2:** Showing the preprocessing steps for raw data collected from local hospitals in Thailand to estimate the reinfection rate of this disease. Those data were obtained from Ranong Hospital at the southern border, Samut Sakhon Hospital at the central area, and Rachaburi at the western border.

**Figure 3:** Schematic representation of SEIRS epidemiological model with dynamic vitals illustrating the compartmental division of population.

**Figure 4:** Sensitivity analysis scatter plots for 1000 sample input parameters.

**Figure 5:** Sobol sensitivity indices for four parameters, beta, sigma, gamma, and mu, are shown in this figure. Total-order sensitivity index (ST) and first-order sensitivity index (S1) are represented in orange and blue colours, respectively. Beta and gamma are critical parameters for the estimation of *R*_0_.

**Figure 6:** Illustration of HFMD confirmed cases from the year 2011 to 2019 throughout Thailand. This figure shows that there is a sharp peak in the number of HFMD cases during the rainy season of each year.

**Figure 7:** Heat map to illustrate HFMD cases from 2011 to 2019 across all the provinces in Thailand. From the figure, we can visualise that the provinces can be grouped into three groups as per the spread of this disease. Bangkok was seen to be the most affected province.

**Figure 8:** Geomapping with clustering of provinces based on the number of infections.

**Figure 9:** Age group of HFMD infected 2019.

**Figure 10:** Shade maps of Thailand entirely with 77 provinces. This map illustrates the severity of HFMD infection spreading and reported over the country in 2019.

**Figure 11:** SEIRS model for provinces in cluster 1 for the years 2011-2019.

**Figure 12:** SEIRS model for provinces in cluster 2 for the years 2011-2019.

**Figure 13:** SEIRS model for provinces in cluster 3 for years 2011-2019.

**Figure 14:** These figures illustrate the predicted and actual HFMD cases in 2020. It is seen that the actual HFMD cases in each clustered province are significantly low compared to the prediction.

**Table 1:** First-order sensitivity index of input parameters (beta, sigma, gamma, and mu) on the basic reproduction number (*R*_0_).

Param	S1	S1 conf	ST	ST conf
Beta	0.467841	0.058418	0.603028	0.063202
Sigma	0.006010	0.009548	0.013932	0.006417
Gamma	0.355064	0.054430	0.493139	0.055598
Mu	0.008948	0.011250	0.018498	0.004292

**Table 2:** Second-order sensitivity index of input parameters (beta, sigma, gamma, and mu) on the basic reproduction number (*R*_0_).

Parameter pairs	S2	S2 conf
Beta/sigma	0.001689	0.073271
Beta/gamma	0.131862	0.109820
Beta/mu	0.005706	0.072474
Sigma/gamma	0.003814	0.013194
Sigma/mu	0.004795	0.012031
Gamma/mu	0.008236	0.071884

**Table 3:** The provinces of Thailand are clustered in 3 clusters based on the number and severity of infections.

Clusters	Infection severity	Provinces
Cluster 1	Low	Lampang, Lamphun, Mae Hong Son, Nan, Phayao, Phrae, Phetchabun, Sukhothai, Tak, Uttaradit, Chai Nat, Kamphaeng Phet, Phichit, Uthai Thani, Angthong, Nakhon Nayok, Nonthaburi, P.Nakhon S.Ayutthaya, Pathum Thani, Sing Buri, Kanchanaburi, Nakhon Pathom, Phetchaburi, Prachuap Khiri Khan, Ratchaburi, Samut Sakhon, Samut Songkhram, Suphan Buri, Chachoengsao, Chanthaburi, Prachin Buri, Sa Kaeo, Trat, Kalasin, Mahasarakham, Roi Et, Bungkan, Loei, Nakhon Phanom, Nong BuaLam Phu, Nong Khai, Sakon Nakhon, Udon Thani, Chaiyaphum, Amnat Charoen, Mukdahan, Yasothon, Chumphon, Krabi, Nakhon Si Thammarat, Phangnga, Phuket, Ranong, Narathiwat, Pattani, Phatthalung, Satun, Songkhla, Trang, Yala

Cluster 2	High	Bangkok

Cluster 3	Average	Chiang Mai, Chiang Rai, Phitsanulok, Nakhon Sawan, Lop Buri, Saraburi, Chon Buri, Rayong, Samut Prakan, Khon Kaen, Buri Ram, Nakhon Ratchasima, Surin, Si Sa Ket, Ubon Ratchathani, Surat Thani

**Table 4:** Reinfection cases were observed at three local hospitals in Thailand.

Year	Reinfection cases	Patients	Percentage
2012	14	383	3.66
2012 to 2013	42	696	6.03
2012 to 2014	91	1151	7.90
2012 to 2015	147	1565	9.39
2012 to 2016	249	2089	11.92

**Table 5:** Estimation of parameters for provinces in cluster 1.

Parameters	2011	2012	2013	2014	2015	2016	2017	2018	2019
*N*	6563521								
*I*_0_	134								
*E*_0_	0	—	—	—	—	—	—	—	—
*T*	12								
*ω*	0.119								
*α*	-0.41	-0.577	0.054	0.337	1.578	-0.256	0.483	-0.083	-0.575
*β*_0_	3.061	1.835	1.964	2.379	1.539	2.007	2.076	2.204	2.186
*σ*	0.739	40.018	2.175	3.015	0.71	11.818	2.836	3.85	4.62
*γ*	3.083	0.919	0.469	0.631	-0.024	0.928	0.384	0.716	0.762
*μ*	-0.331	1.261	0.81	1.067	0.398	1.151	0.996	1.033	1.065
*R*_0_	15.261	3.877	1.829	2.984	0.369	3.802	2.121	3.038	3.246

**Table 6:** Estimation of parameters for provinces in cluster 2.

Parameters	2011	2012	2013	2014	2015	2016	2017	2018	2019
*N*	779326								
*I*_0_	39								
*E*_0_	0	—	—	—	—	—	—	—	—
*T*	12								
*ω*	0.119								
*α*	-0.512	-0.781	0.879	0.813	1.438	-0.001	1.115	0.998	-0.317
*β*_0_	4.749	4.821	1.488	1.216	0.68	1.388	1.522	1.673	1.812
*σ*	1.103	74.438	0.761	4.683	4.253	29.975	2.134	1.436	7.488
*γ*	5.861	3.539	-0.623	-0.052	-0.825	0.552	-0.111	-0.099	0.624
*μ*	-0.477	2.98	0.947	0.846	1.066	0.877	0.797	0.717	1.036
*R*_0_	45.07	30.221	0.215	0.818	0.131	1.927	0.761	0.689	2.643

**Table 7:** Estimation of parameters for provinces in cluster 3.

Parameters	2011	2012	2013	2014	2015	2016	2017	2018	2019
*N*	3604332								
*I*_0_	107								
*E*_0_	0	—	—	—	—	—	—	—	—
*T*	12								
*ω*	0.119								
*α*	-0.633	0.264	0.936	0.271	-0.435	-0.194	1.104	-0.177	-0.092
*β*_0_	2.802	0.634	0.825	1.896	2.022	1.632	1.572	2.16	1.907
*σ*	0.622	83.55	2.907	5.728	1.752	23.559	2.208	2.916	3.074
*γ*	2.279	0.34	-0.578	0.616	0.368	0.674	-0.382	0.73	0.384
*μ*	-0.174	0.131	0.891	1.033	0.866	1.054	1.055	0.84	0.917
*R*_0_	8.189	0.298	0.198	2.649	1.67	2.699	0.715	2.632	1.91

**Table 8:** Calculation of *R*^2^.

Clusters	*R* ^2^
Cluster 1	0.63
Cluster 2	0.777
Cluster 3	0.756

## Data Availability

Data used in this experiment are available in doi:10.6084/m9.figshare.13238966.v1.

## Abbreviations

BoE: Bureau of Epidemiology
HFMD: Hand, foot, and mouth disease
SIR: Susceptible-infectious-recovered
SEIR: Susceptible-exposed-infectious-recovered
SEIRS: Susceptible-exposed-infectious-recovered-susceptible
SEIQR: Susceptible-exposed-infectious-quarantined-recovered.
